This article has been retracted.

# Clinical Treatment Analysis and Imaging Study of Patients with Acute Angina in Cardiovascular Medicine

**DOI:** 10.1155/2021/1458621

**Published:** 2021-09-27

**Authors:** Peng Li, Li He

**Affiliations:** Peoples Hospital of Tongcheng City, Xianning 437400, Hubei, China

## Abstract

With the accelerating pace of life, increasing stress and unhealthy diet make cardiovascular disease one of the important diseases that endanger human health, among which the incidence of acute angina is gradually increasing. At present, there are many clinical treatment studies on acute angina pectoris, but the relevant imaging analysis is very lacking. In order to study the clinical treatment of patients with acute angina pectoris and analyze the relevant medical images, to arrive at a more effective treatment method, this article launched an in-depth study. First, we selected 88 patients with acute angina in a hospital as the research object and randomly divided them into a control group (*n* = 44) and an experimental group (*n* = 44) Yan et al. (2020). The control group was treated with conventional acute angina pectoris drugs, while the experimental group was treated with clopidogrel on this basis. The two groups were treated at the same time, and the treatment time lasted for 3 months. Then, the risk factors of the two groups of patients were analyzed, and the differences were statistically significant (*P* < 0.05). Then, the medical images of the two groups of patients were analyzed, and the diastolic blood pressure, systolic blood pressure, and coronary artery stenosis were compared before and after treatment. After treatment, the diastolic blood pressure and systolic blood pressure of the experimental group were 88.31 ± 3.15 mmHg and 125.63 ± 4.16 mmHg, respectively. The proportion of patients with zero-vessel disease and single-vessel disease in the experimental group increased to 15.91% and 56.82%. The treatment plan received by the experimental group patients had a better improvement effect. Finally, the clinical efficacy was compared. The total effective rates of the control and experimental groups were 72.7% and 88.6%, respectively. This shows that the treatment method adopted by the experimental group of patients has a better curative effect and is worthy of clinical promotion.

## 1. Introduction

### 1.1. Background Significance

The morbidity of cardiovascular diseases occupies a major position in the world, and they are still on the rise. Among them, acute angina pectoris is more common clinically and is one of the main factors that induce coronary heart disease [1, 2]. At present, medical imaging has important clinical significance in guiding and planning before treatment, tracking and positioning during treatment, and prognostic progress [3]. Therefore, analyzing the clinical treatment of patients with acute angina in cardiovascular medicine from the perspective of medical imaging has important reference significance for clinical efficacy.

### 1.2. Related Work

Cardiovascular disease has always been the focus of medical research due to its high morbidity and mortality. To compare the incidence of cardiovascular disease in morbidly obese diabetic patients and non-diabetic patients, Pontiroli et al. collected medical records of obese patients who received LAGB or medication from 1995 to 2001. They matched the patient's age, gender, BMI, and blood pressure [4]. Through an extensive literature search, Mohammad et al. collected, summarized, and classified existing information on cardiovascular disease mortality and morbidity in different populations in Bangladesh [5]. Their research conclusions have reference significance for the treatment of cardiovascular diseases, but the patient data they refer to are from a long time ago. Acanfora et al. allowed forty-five patients (42 males and 3 females) suffering from chronic stable angina pectoris and coronary artery disease recorded by angiography to take different doses of single-dose lercanidipine at 3 hours and 8 hours after administration. The effectiveness of anti-ischemia and anti-angina pectoris was evaluated by bicycle exercise test [6]. Medical imaging is of great significance to clinical treatment, so it is the focus of attention. Adali et al. proposed to apply the two models of joint independent component analysis (jICA) and transposed independent vector analysis (tIVA) to the fusion of multimodal medical image data [7]. Their research is innovative, but their method is too complicated to promote.

### 1.3. Innovative Points in This Paper

In order to improve the clinical efficacy of acute angina pectoris in cardiovascular medicine, provide data reference for the treatment of related diseases, and improve the quality of life of patients, this article analyzes the clinical treatment of acute angina pectoris from the perspective of medical imaging [8]. The innovations of this study are as follows: (1) grouping treatment of patients with acute angina in the cardiovascular department of a hospital, comparing the risk factors of the two groups, and obtaining statistically significant risk factors; (2) analyzing the medical images of the two groups of patients, performing coronary angiography and electrocardiogram detection, comparing the diastolic blood pressure, systolic blood pressure, and coronary artery stenosis before and after treatment, and concluding that the treatment plan of the experimental group has better improvement; and (3) comparing the clinical efficacy, it is found that patients can have a better therapeutic effect by adding an appropriate amount of clopidogrel on the basis of conventional treatment.

## 2. Angina Pectoris Treatment and Imaging Analysis

### 2.1. Cardiovascular Diseases

#### 2.1.1. Risk Factors of Cardiovascular Diseases

Cardiovascular diseases include myocardial infarction, angina pectoris, and coronary atherosclerosis [9]. At present, the main risk factors for cardiovascular disease recognized internationally include age, family history, hypertension, dyslipidemia, obesity, unhealthy diet and rest, diabetes, smoking, and lack of exercise [10]. Many of these risk factors can be improved through our own efforts.

Blood pressure level and cardiovascular disease have a close relationship independent of other risk factors. The risk of stroke and myocardial infarction increases with blood pressure [11]. Smoking can induce arrhythmia through many mechanisms, leading to heart deterioration.

Dyslipidemia is mainly manifested as high-density total cholesterol, which is closely related to the risk of coronary heart disease. Even if the sex is different, there is a strong negative correlation between high-density lipoprotein cholesterol and coronary heart disease. For every 1% decrease in total cholesterol, the risk of coronary heart disease will be reduced by 3% [12]. The long-term accumulation of excessive fat in the body can cause metabolic disorders and affect the system that regulates inflammation.

#### 2.1.2. Risk Prediction and Evaluation Indicators for Cardiovascular Diseases

Abnormal blood lipid metabolism will directly affect the functional damage of vascular endothelial cells. The endothelial tissue covers the entire surface of the vascular cavity, regulates the vascular movement function, adjusts the stability of blood flow, reshapes the vascular structure, and plays a good protective barrier role. The path leading to lipid metabolism disorders in the blood is mainly the oxidized low-density lipoprotein path. Endothelial dysfunction caused by hypercholesterolemia can be corrected by adjusting the level of low-density lipoprotein cholesterol [13]. Since the increase of active substances such as norepinephrine and amino acid in the body can cause the dysfunction of vascular endothelial function, the damage of endothelial function caused by hyperlipidemia may be a potential cause of hypertension, hyperlipidemia, and other cardiovascular diseases.

The blood total cholesterol level is closely related to the blood pressure level. Abnormal blood lipid metabolism will affect the lipid structure of the cell membrane and then affect the calcium ion transport process of the cell membrane, which may be involved in the occurrence of hypertension and other diseases. Low-density lipoprotein cholesterol, serum total cholesterol, and triglycerides in patients with hypertension may affect the transparency of cell membranes that are closely related to the influx of calcium ions [14].

Other serum biochemical markers such as high-density lipoprotein cholesterol and chylomicrons are closely related to low-density lipoprotein cholesterol and are also related to the risk of cardiovascular disease. The pathological changes in the early stage of atherosclerosis refer to the deposition of lipid particles rich in low-density lipoproteins under the arterial endothelium, thereby increasing the concentration of low-density lipoprotein cholesterol in the blood circulation. This is a necessary condition for the formation of atherosclerosis and an important cause of the disease.

#### 2.1.3. Treatment and Prevention of Cardiovascular Diseases

Cardiovascular diseases have different symptoms, and their specific treatment methods are also different. However, overall, all cardiovascular diseases can be treated by the following treatment methods. First of all, the patient's mentality must be kept in a good state, with not too much emotional ups and downs. The second is to carry out appropriate exercises in a targeted manner, reasonably arrange the time and amount of exercise to maintain the health of the body, and improve immunity. Third, we must control risk factors, maintain normal blood pressure, control diabetes, quit smoking, and have a healthy diet. The last is drug treatment and surgical treatment. Different cardiovascular diseases require targeted drug treatment and surgical treatment to relieve symptoms and improve prognosis.

The prevention of cardiovascular disease includes primary prevention and secondary prevention. The so-called one-time prevention refers to prevention before the onset, that is, to prevent the occurrence of the disease. The so-called secondary prevention is to reduce the risk of recurrence and prevent it from happening again.

Blood vessels tend to contract and spasm in the cold winter, and the blood supply is insufficient, which may cause embolism, so care must be taken to keep warm. High-risk patients can receive effective antithrombotic therapy and can take aspirin for a long time under the guidance of a doctor [15]. Patients should pay attention to proper warm-ups during morning exercises, arrange exercises reasonably, and avoid sudden increases in nerve excitement to induce diseases. An unhealthy lifestyle has a direct impact on the recovery and prognosis of the disease. Therefore, it is necessary to manage total food intake, adjust diet structure, quit smoking, and drink less alcohol.

### 2.2. Treatment of Acute Angina

#### 2.2.1. Causes of Acute Angina Pectoris

The direct cause of angina pectoris is the absolute or relative insufficiency of myocardial blood supply. Therefore, various reductions in myocardial blood supply and an increase in oxygen consumption will induce angina. The insufficient blood supply to the myocardium is mainly caused by coronary heart disease [16].

Fat deposits in blood vessels form plaques. Plaques in the coronary arteries can cause coronary heart disease. The coronary arteries continue to deposit fat and slowly form plaques [17]. Plaque causes the stenosis and hardening of the coronary arteries themselves, and blood clots block the coronary arteries, which can cause angina.

Angina pectoris can also be caused by physical labor, large mood swings, fear, and cold. Typical angina pectoris usually occurs under the same working conditions, and angina pectoris that occurs in a quiet state is the result of coronary artery spasm. The mechanism of pain during myocardial ischemia may be caused by certain products in myocardial anaerobic metabolism that stimulate the heart to the end of the heart nerve, which often spreads across the surface nerves of the skin in the same spinal cord, causing pain.

#### 2.2.2. Diagnosis of Acute Angina Pectoris

The diagnosis of acute angina must consider its predisposing factors, such as excessive physical work and large mood swings. At the onset, the patient has severe pain in the chest. The range of pain is generally the size of the palm and fist. The main types of pain are burning pain, squeezing pain, and clamping pain. The duration of pain in patients is generally 3 to 5 minutes, and there is short-term pain within 1 minute [18]. If the pain is relieved after taking nitroglycerin, it can be diagnosed.

The diagnosis of angina pectoris needs to be distinguished from the symptoms of acute myocardial infarction, chest soft tissue lesions, and cardiac neurosis. The chest pain is severe and the oral administration of nitroglycerin has not been relieved, so it is necessary to check the electrocardiogram and myocardial enzymes to detect the possibility of acute myocardial infarction [19].

If the location of the pain is fixed and there is obvious tenderness, which will aggravate the pain during thoracic exercises, it is necessary to consider whether it is related to chest soft tissue lesions. The chest pain lasts for a few seconds or several hours or days. The nature of the pain is dull pain or difficulty in breathing, and the location is almost little. In most cases, the pain is not at the time, but after exercise. It will continue after taking nitroglycerin, and it will be relieved after a period of time. During the period, upset and anxiety will also occur, which is mainly considered to be cardiac neurosis.

#### 2.2.3. Treatment of Acute Angina Pectoris

The treatment of acute angina pectoris generally needs to be carried out in accordance with the following principles: first, determine the inducing cause of angina pectoris, treat risk factors, perform appropriate exercise, and improve lifestyle. Then, start to take aspirin according to the doctor's advice and take nitroglycerin to improve symptoms; when the number of attacks exceeds two times a week, calcium channel blockers should be added to nitroglycerin. If angina is not controlled, long-acting nitrates can be added [20]. However, it should be noted that the frequency and severity of angina pectoris and the type of pain must be taken into consideration when using the abovementioned drugs. If the combination of two or more drugs has not reduced the number of angina pectoris, coronary angiography should be considered for surgical treatment.

Common drugs can be divided into anti-platelet aggregation drugs, calcium channel blockers, nitrate drugs, and angiotensin-converting enzyme inhibitor drugs [21]. Anti-platelet aggregation drugs inhibit platelet aggregation and exert anti-platelet effects. Calcium channel blockers can dilate coronary blood flow and reduce blood pressure and myocardial oxygen consumption. Nitrate drugs can mainly increase the blood supply of ischemic myocardium. Angiotensin-converting enzyme inhibitor drugs can reduce the symptoms of cardiac hypertrophy and thickening of blood vessel walls.

Surgical treatment includes percutaneous coronary intervention and coronary artery bypass grafting, collectively referred to as coronary revascularization treatment. The prerequisite for vascular reconstruction treatment is that the effect of drug treatment cannot satisfy the patient. The results of non-invasive examination show that most of the myocardium is already at risk. The operation has a high success rate, and the patient can accept the relevant risks. Percutaneous coronary intervention can dilate blood flow, eliminate or reduce angina pectoris, and improve electrocardiogram. Coronary artery bypass grafting can improve the prognosis, and it is also effective for intermediate-risk and even high-risk patients.

### 2.3. Medical Imaging Technology

#### 2.3.1. Types of Medical Imaging

CT images can be used for target positioning and precise radiotherapy plans for clinical cases. During treatment, patients can be treated with radiotherapy according to the plan. The prerequisite work of making the plan is to realize the automatic segmentation of the target organs in clinical CT images. The plan needs to be based on the HU value information of the CT image, so it is necessary to locate the target organ target area, outline the relevant organ at risk, use software to simulate the radiotherapy process, and form a radiation dose distribution curve on the CT image [22]. CT images are relatively reliable for obtaining the location, number, and size of the lesion area. In order to get proper diagnosis and treatment, it is necessary to combine the experience of clinicians and comprehensive analysis of other clinical medical images.

4DCT imaging technology can acquire imaging targets at different moments and observe changes in the shape and position of target organs [23]. In the process of clinical radiotherapy, the deformation and movement of other related organs and tissues, as well as the errors caused by changes in the positions of various systems and organs, will inevitably occur, and the endangered organs related to the target area of the target organ tumor may be out of irradiation. Therefore, it is necessary to collect real-time image information for image-guided radiotherapy. CBCT can use different ways to track target organs, which improves the accuracy of image-guided radiotherapy.

#### 2.3.2. Classification of Medical Image Segmentation Technology

Medical image segmentation technology can be divided into two main categories. One is a method that does not use prior information, such as differential operator edge detection algorithm, threshold method, region expansion method, morphological segmentation method, and so on [24]. This type of method has low robustness and accuracy when realizing target area division and poor versatility. It needs to be used in combination with other methods based on prior information. Another type of method is a segmentation method based on prior information. This type of method has higher computational complexity and segmentation accuracy for a specific organization, but its robustness is very low and it is prone to false segmentation. Therefore, in actual clinical applications, it is necessary to comprehensively apply the two methods to obtain better segmentation results.

The discontinuity of the edge points of the image can be detected by the derived method [25]. The image segmentation algorithm uses the zero-crossing point information of the first derivative or the second derivative of the image to find the edge area. Edges are mainly divided into two types: step edges and roof-like edges. The gray values of the pixels perpendicular to the edge of the step are significantly different. The roof edge is the transition point from the increase in the gray value to the decrease. The second derivative of edge detection algorithm includes Gauss–Laplace edge detection operator and Canny edge detection algorithm [26]. The Laplace value of the Gaussian function is shown in the following formula :

(1) $$\begin{array}{c} \frac{1}{2\pi \sigma^{2}}\left(\frac{x^{2}+y^{2}-\sigma^{2}}{\sigma^{4}}\right)\exp\left(-\frac{x^{2}+y^{2}}{2\sigma^{2}}\right), \end{array}$$

where *G*(*x*, *y*, *σ*) represents a two-dimensional Gaussian function.

The threshold method divides the image into multiple subareas according to the gray level by selecting one or more thresholds. Each subregion has specific similarities, and different subregions have different properties. This method is simple to calculate, efficient, and widely used. Threshold segmentation is mainly divided into global threshold segmentation method and local threshold segmentation method. The methods for determining the best global threshold generally include experimental methods, histogram methods, and the minimum error method assuming that the gray distribution of the background area and the target area conforms to the normal distribution. If all pixels cannot use a threshold to properly segment the image, the local threshold segmentation method can be used to segment the image. The process of threshold segmentation is shown in the following formula :

(2) $$\begin{array}{c} g_{K}\left(x,y\right)=\left\{\begin{array}{cc} 1, & \mathrm{if,}\\ 0, & \mathrm{else,} \end{array}\right)\;f\left(x,y\right)\geq K, \end{array}$$

where *f*(*x*, *y*) is the gray value at the image point (*x*, *y*) and the gray range is [0,1].

#### 2.3.3. Technical Issues of Medical Image Segmentation

In the process of acquiring or sending, medical images are easily disturbed by various noises, destroying the integrity of the image, and unable to obtain more refined or meaningful feature information. Different imaging sensors have inconsistent signal acquisition principles, and different modal images have many kinds of noise, but each modal image will be affected by the main noise interference [27].

Part of the volume effect is due to the limited spatial resolution of imaging equipment, and individual units contain multiple types of tissues and organs. Therefore, the gray values of the boundaries of various tissues and organs are very close, and the boundaries of tissues and organs cannot be distinguished, so the image segmentation work becomes very difficult.

The non-uniformity of image intensity usually refers to the grayscale changes of the same type of tissue, including the grayscale range of the entire image. Multiple pixel areas with different gray levels are prone to exist in the same lesion area, and pixel classification errors may occur. The slight unevenness in the MRI image is mainly reflected in the problem of the offset field, which needs to be smoothed by the offset field correction algorithm before segmentation.

## 3. Experiments on Clinical Treatment and Imaging Analysis of Patients with Angina Pectoris

### 3.1. Research Objects

A random selection of 88 patients with acute cardiovascular angina who were admitted to a hospital from January 2018 to December 2018 were the subjects of the study. They were randomly divided into a control group and experimental group, with 44 patients in both groups. There were 18 males and 26 females in the control group, aged 38–65 years old, with an average age of (54.29 ± 2.15) years, and there were 24 males and 20 females in the experimental group, aged 40–68 years old, with an average age of (58.34 ± 2.67) years old.

Inclusion criteria were as follows: sudden suffocation pain in the left chest; the range of pain is generally the size of the palm and fist; and T wave inversion appeared on the lead without T wave inversion and exceeded 2 mm.

Exclusion criteria were as follows: incomplete basic data and medical history records; patients who did not receive cardiac color Doppler ultrasound and coronary angiography during hospitalization; patients with acute myocardial infarction; and patients with liver and kidney dysfunction.

### 3.2. Methods

The age, gender, smoking, and alcoholism of the two groups of patients, past medical history, and predisposing factors were collected. The criterion for a positive smoking history is to smoke at least one cigarette a day and smoke continuously for more than one year. Past medical history includes type 2 diabetes, hypertension, coronary heart disease, and dyslipidemia.

The patients in the control group took conventional angina pectoris drugs orally and selected different drugs such as receptor blockers and aspirin enteric-coated tablets according to the specific conditions of the patients. In the experimental group, clopidogrel was added to the conventional treatment. The treatment of the two groups of patients was 1 month as a course of treatment and continued treatment for 3 courses.

### 3.3. Evaluation Criteria and Statistical Methods

The evaluation standard is based on the evaluation standard of acute angina pectoris, and the treatment results are divided into three levels: markedly effective, effective, and ineffective. Markedly effective means that the patient's ECG is normal at rest. Effective means that the patient's ST-segment declines and rises more than 0.5 mV in the resting state, but it still does not reach the normal level. Invalid means that the patient's ECG at rest does not meet the above standards. The total effective rate of curative effect is calculated as shown in the following formula:

(3) $$\begin{array}{c} P=\frac{\left(X+Y\right)}{N}\times 100\%, \end{array}$$

where *X*, *Y*, *N* represent the number of markedly effective patients, the number of effective patients, and the total number.

Coronary angiography was performed on the two groups of patients, and the lesion location and severity of the coronary vessels were recorded. According to the number of lesions, the lesions can be divided into zero-vessel disease, single-vessel disease, double-vessel disease, and multi-vessel disease.

The relevant information and data of the patients in this study were statistically analyzed using SPSS24.0 statistical software, and the *t*-test and *x*^2^ test were performed. *P* < 0.05 was considered as a statistically significant difference.

## 4. Discussion on Comparison of Clinical Treatment Effects and Imaging Analysis

### 4.1. Comparison of Risk Factors

####  4.1.1. Risk Factors of Data Calculation

Before the start of treatment, the risk factors of the two groups of patients were compared. First, based on the number of people, list the risk factors of the data calculation type. This study selected six factors: gender, hypertension, type 2 diabetes, smoking, alcoholism, overwork, and mood swings, for analysis. The comparison results are as follows.

As shown in Figure 1, there are differences in the number of risk factors between the control group and the experimental group. After calculation, the difference between the proportion of males (40.9% and 54.5%) and smoking history (18.2% and 29.5%) was statistically significant (*P* < 0.05). Among them, the three factors of hypertension, alcoholism, and mood swings all differed by only one person. The difference was statistically insignificant.

#### 4.1.2. Risk Factors of Measurement Data

Before the start of treatment, the risk factors of the two groups of patients were compared, and the risk factors of the measurement data type were also compared. This study selected 6 factors of white blood cell count (WBC), renal function (Cr), fasting blood glucose (FBG), total cholesterol (TC), low-density lipoprotein (LDL-C), and triglycerides (TG) for comparison, and the comparison results are as follows.

As shown in Table 1, the experimental results of the control group are higher than those of the experimental group, and the difference is statistically significant (*P* < 0.05).

### 4.2. Medical Imaging Analysis

#### 4.2.1. Diastolic and Systolic Blood Pressure

After 3 months of treatment, diastolic blood pressure and systolic blood pressure were measured for the patients in the control group and the experimental group and compared with the data before treatment to observe the changes of related indicators under different treatment methods. The diastolic blood pressure before and after treatment is represented by D1 and D2, and the systolic blood pressure before and after treatment is represented by S1 and S2.

As shown in Figure 2, after 3 months of treatment, the diastolic and systolic blood pressures of the two groups were significantly lower than before treatment. After treatment, the diastolic blood pressure and systolic blood pressure of the control group were 94.38 ± 3.27 mmHg and 131.37 ± 4.38 mmHg, respectively. This indicates that the treatment program received by the experimental group has a better effect on improving the two indicators of diastolic and systolic blood pressure.

#### 4.2.2. Results of Coronary Angiography

After 3 months of treatment, patients in the control group and the experimental group were subjected to coronary angiography and compared with the number of coronary artery stenosis before treatment to observe the changes in the number of coronary artery stenosis under different treatment methods. Zero-vessel disease, single-vessel disease, double-vessel disease, and multi-vessel disease are represented by B0, B1, B2, and B3, respectively. The control group and experimental group before and after treatment are represented by C1 and C2 and E1 and E2.

As shown in Figure 3, before and after treatment, the number of coronary artery stenosis in the control group and the experimental group changed. The proportion of zero-vessel disease and single-vessel disease became larger. After treatment in the experimental group, the proportion of zero-vessel disease and single-vessel disease increased from 4.55% and 45.45% to 15.91% and 56.82%. This indicates that the treatment program received by the experimental group has a better effect on improving coronary stenosis.

### 4.3. Comparison of Clinical Efficacy

After systematic treatment, the treatment methods of the two groups of patients have produced certain effects. We compare the clinical efficacy of the control group and the experimental group and calculate its total effective rate. The comparison results are as follows.

As shown in Figure 4, the proportions of markedly effective, effective, and ineffective clinical efficacy of the control group were 25%, 47.7%, and 27.3%, respectively. After calculation, the total effective rates of the control group and experimental group were 72.7% and 88.6%, respectively. This shows that the treatment method used by the experimental group of patients has got a better effect.

## 5. Conclusions

Cardiovascular diseases are caused by heart and vascular diseases, and acute angina pectoris is one of the common cardiovascular diseases. The main internationally recognized risk factors for cardiovascular disease include high blood pressure, dyslipidemia, obesity, unhealthy diet and rest, diabetes, smoking, and alcoholism. For the treatment of acute angina pectoris, we must first determine the exact cause of angina pectoris and the risk factors that may exist during treatment and then start taking the medicine as prescribed by the doctor. If the combination of two or more drugs has not reduced the number of angina pectoris, coronary angiography should be considered for surgical treatment.

Medical imaging has important clinical significance in guiding and planning before treatment, tracking and positioning during treatment, and prognostic progress. However, in the process of acquiring or sending, medical images are easily disturbed by various noises, destroying the integrity of the image.

Among patients with acute angina pectoris, the differences in risk factors such as the proportion of men, smoking history, fasting blood glucose, total cholesterol, low-density lipoprotein, and triglycerides were statistically significant. By comparing the diastolic blood pressure, systolic blood pressure, coronary artery stenosis, and the clinical efficacy of the two groups of patients, it was found that the addition of appropriate clopidogrel on the basis of conventional treatment in patients with acute angina can improve the efficacy.

## Figures and Tables

**Figure 1:** Comparison of risk factors (count data) between the two groups.

**Figure 2:** Comparison of indicators before and after treatment between the two groups.

**Figure 3:** Comparison of coronary artery stenosis before and after treatment between the two groups.

**Figure 4:** Comparison of clinical efficacy between the two groups of patients.

**Table 1:** Comparison of risk factors (measurement data) between the two groups of patients.

Risk factors	Control group	Experience group	*P*
WBC (10^9^/l)	12.14 ± 3.25	11.83 ± 3.79	0.071
Cr (*μ*mmol/l)	70.21 ± 13.87	71.54 ± 15.35	0.524
FBG (mmol/l)	6.11 ± 0.98	5.28 ± 0.84	≤0.001
TC (mmol/l)	4.58 ± 1.16	4.26 ± 1.08	0.021
LDL -C (mmol/l)	3.27 ± 0.94	2.59 ± 0.72	≤0.001
TG (mmol/l)	3.22 ± 0.98	2.13 ± 0.69	≤0.001

## Data Availability

The data that support the findings of this study are available from the corresponding author upon reasonable request.
